# Robotic and Microrobotic Tools for Dental Therapy

**DOI:** 10.1155/2022/3265462

**Published:** 2022-02-18

**Authors:** Chen Cheng, Xue Yinan, Xie Zongxin, Shi Lei, Xue Yanan, Yang Yanli

**Affiliations:** ^1^Stomatology Hospital, School of Stomatology, Zhejiang University School of Medicine, Zhejiang Provincial Clinical Research Center for Oral Diseases, Key Laboratory of Oral Biomedical Research of Zhejiang Province, Cancer Center of Zhejiang University, Hangzhou 310006, China; ^2^Biological Science, College of Chemistry and Life Sciences, Zhejiang Normal University, Jinhua 321000, China; ^3^Stomatology Hospital, Zunyi University School of Medicine, Zunyi 563000, China; ^4^Department of Plastic Surgery, Sir Run Run Shaw Hospital, Zhejiang University of Medicine, Hangzhou 310016, China

## Abstract

Robotic and microrobotic tools such as dental operating microscopes and dental endoscopes are being used extensively in dental therapy, which have a significant impact on dental therapy and education. Herein, this paper reviews the state of the art of robotic and microrobotic tools for dental therapy. This article starts with a brief introduction of current robotic and microrobotic tools for dental therapy and then displays their applications in various dental problems; strengths and weaknesses are also surveyed. Lastly, the conclusion and outlook are discussed, referring to the emerging dental clinic problems and demands. This review is expected to provide guidelines for the therapeutic application of robotic and microrobotic tools and to promote the development of robots in dentistry.

## 1. Introduction

From a surgery perspective, the main symbol of the 21st century is the progression of robotic surgery. Robots have developed rapidly in the field of medicine. They are mainly used to assist doctors to complete minimally invasive surgery or reach positions that are difficult to reach by hands. Robotics is a disruptive technology that will change diagnostics and treatment protocols in dental medicine. A robot device acts as a computer interface between the operator and the instrument. In some cases, this ensures that some surgeons who struggle with “straight” videoscopic operations face fewer technical challenges than traditional methods. The use of robotic tools influences what we can do evidently. For a long time, dental therapy has been hampered by the tiny space available in the mouth, making it difficult to see the surgical field. Unfortunately, robots are not used as extensively in dentistry as in medicine [1]. Few promising robotic systems are not yet available to dentists. Robotic therapy is developing slowly in dental medicine. Recent research shows that only a few authors with a dental or medical background were involved in articles about robots [2]. This omission truly harms the development and promotion of dental robots. Under these circumstances, robotic engineers have difficulty understanding the needs of dentists. Robotic and microrobotic tools have started to help dentists as magnification devices in therapy, but they are still difficult to automate. There is an urgent need to guide engineers to finally transform these robotic and microrobotic tools into robots. The development of microscopes toward the end of the 16th century started the use of robotic tools [3]. Robotic and microrobotic tools, including dental operating microscopes and dental endoscopes, are now often used [4, 5]. Robotic and microrobotic tools bring a series of advantages: they improve the dentists' operating position and prolong the dentists' professional life; the built-in light source illuminates the affected area and provides a clear surgical field of vision; the adjustable multiple magnifies the affected area and makes the structure of teeth visible, which provides the possibility for the accuracy of the operations [6, 7]. Dental microscopes were first used in endodontics and then widely used in various oral subspecies [6–8]. It seems that robotic and microrobotic tools can meet the needs of dentists, which robots cannot do. Nowadays, Three-Dimensional Robotic Digital Microscope is playing an implant role in neurosurgery [9]. A new robotic microscope is also reported in 2020 [10]. Robotic endoscopes are also in service in the gastrointestinal system [11]. These advanced robotic tools are one step closer to full automation. However, these robotic tools are still relatively low-end in dental treatment.

The utilization and development of robotic and microrobotic tools in endodontics and other oral subspecies will be discussed in depth in this study. The review will also focus on the needs of the dentists and current issues with robotic and microrobotic tools. We want to guide the development of dental robots according to the applications of these robotic and microrobotic tools.

## 2. Robotic and Microrobotic Tools

Robotic and microrobotic tools working as robotic imaging systems for dental clinical treatment include dental operating microscopes and dental endoscopes, as shown in Figures 1(a) and 1(b). The robotic system of endoscopes is shown in Figure 1(c).

### 2.1. Dental Operating Microscopes

Dental operating microscopes (DOMs) are stereomicroscopes. The microscope's left and right light paths provide different object angles to achieve a magnified three-dimensional image. The zoom system magnifies the image through multiple groups of lenses according to the selected magnification. A dental operating microscope can provide 2–30 times magnification, which can be adjusted according to doctors' demands [8]. A microscope can usually be used as the eye of a robot. Robots usually appear to complete a minimally invasive surgery, so microscopy is an indispensable part of robots. Previous studies show that the use of DOM among endodontics has increased significantly since the early 1990s; a survey in 2008 showed the frequency of DOM use by endodontics to be 90% [12]. Thus, the DOM is an integral tool in today's endodontic practice, which helps to optimize the visualization of the tooth and its substructures [6, 13]. The benefits of DOM in nonsurgical and surgical endodontic procedures have been reported. Advantages include facilitating access preparation [14]; locating canal orifices [15]; enhancing fine motor skills [16]; improving the ability to examine, clean, and shape the complex canal anatomy; removing and bypassing separated instruments; detecting fracture lines; assisting in obturation; and improving surgical techniques [17–19]. Despite its advantages, DOM is far from an ideal magnifying tool for dental procedures. Currently, dental endoscopes are regarded as an alternative to microscopy.

### 2.2. Dental Endoscopes

Endoscopes are standard medical devices composed of an intraoral camera, an endoscope probe, and a computer. At present, an endoscope is one of the common tools for the application of microrobots. The common structure of an endoscope is shown in Figure 2. Despite the availability of these diagnostic devices, however, the observation of collateral root canals and fractures near the deep root canal area, the root apex, remains difficult. Moreover, dental operating microscopes only allow assessing areas close to the root canal entrance, and tomography does not provide the resolution required to identify fine structures and cannot be used under endodontic treatment. In contrast, endoscopes can allow high-resolution and almost noninvasive observation inside the root canals under treatment, and they are under active research for various applications [20]. Previous studies have shown that dental endoscopes are a popular device to remove things falling into the sinuses, trachea, esophagus, or other cavities [21]. Thus, dental endoscopy has also been reported for implant surgery [22]. Historical studies have shown that endoscopy can assist periodontal surgery [23], joint surgery [24], bone marrow cavity observation [25], wound repair [26, 27], osteotomy [28], salivary lithotripsy [29, 30], biopsy [31, 32], polypectomy [33], stereotactic radiotherapy [34], tumor removal [35], and even nerve visualization [36]. It also has certain significance for oral distance teaching and telediagnosis [37]. Endoscopes can realize the microtransportation of light-curing materials, compare the effect of apical surgery, explore root canals, observe dental pulp, and realize root canal visualization [38–40]. In 2018, an endoscopic system based on an intraoral camera and image processing was reported [41]. This system is the first step to facilitating the observation of fine structures by intraoral cameras.

## 3. Robotic and Microrobotic Tools in Dental Treatment

### 3.1. Robotic and Microrobotic Tools in Endodontics

Endodontic therapy includes treating the infected dentin, enamel, and pulp of a tooth to remove the infection and the pain it causes. Successful endodontic therapy relies on mechanical and chemical cleansing of the entire infected space and its complete obturation with an inert filling material [42–44]. The different morphologies of the tooth structure lead to the unpredictable shape of the root canal system. In traditional endodontic therapy, dentists find the root canal by freehand and mouth mirrors. Although there are various auxiliary instruments, the chance of missing root canals is still hard to avoid. For example, the second mesiobuccal canal (MB2) of maxillary molars has a high probability of existence, but it is not easy to locate with the naked eye [45]. To increase the success of endodontic therapy, Pro. Apotheker and Jako invented the dental microscope in 1978. The first dental microscope was born in 1981 and is named dentiscope [46]. After 1993, dental microscopes became popular and were widely used in endodontic therapy. Currently, microrobotic tools are widely used in endodontic therapy [47].

#### 3.1.1. Identify Caries and Cracked Teeth

The enamel will show early decay, microleakage, and a lack of dentin and enamel structural integrity at extreme magnification levels. Caries decayed in teeth, whose sensitivity of diagnosis was significantly greater when magnification was used, as shown in Figure 3(a). Microrobotic tools also provide support for more precise fillings. In 2015, a miniature probe for delivery and monitoring of a photopolymerizable material was invented [48]. In addition, dentists diagnose cracked teeth by symptom-driven methods, as usual. The lack of visual confirmation always delays the diagnoses and therapies. Microleakage under a microscope will help dentists diagnose cracked teeth, as shown in Figures 3(b) and 3(c). An in vitro study showed that a fabricated root canal endoscope could facilitate detailed visualization of the apical foramen of a curved root canal and the fracture lines of the inside wall of a root canal [49].

#### 3.1.2. Root Canal Treatment

*(1) Location of Root Canals*. Determining the location of root canals is the most critical and challenging step of root canal treatment. Missing canals more easily occur without microrobotic tools [50]. These missed or untreated canals were full of necrotic tissue and bacteria, leading to chronic symptoms and nonhealing periapical lesions. Root canal location is facing severe challenges because of the complexity of the root canal system. The ML canal in MB roots of maxillary molars can be tough to locate. ML canal detection was increased by adding microrobotic tools from 51% to 82% in 39 test teeth [51]. The magnification of the operating field provided by the microscope and dental loupes is an essential factor in successfully locating the MB2canal, as shown in Figures 3(f) and 3(g) [52]. Figure 3(e) shows P2 of the anterior teeth, and Figure 3(h) shows ML2 of the posterior teeth. Keles et al. reported a comparative study on the accuracy of an endoscope to detect root canal anastomoses in mandibular molar teeth with microcomputed tomography. Divergence points located on the inner wall of main mesial root canals were undetectable under magnification via DOM, while endoscopic examination could detect 23.4% of them at the coronal halves of canals [53].

*(2) Root Canal Preparation*. The ideal endodontic treatment is based on adequate root canal preparation and suitable filling with inert filling materials. Root canal treatment should obtain proper root canal shape, with efficient cleaning performed before filling. However, factors such as root canal calcification and root canal variation and the anatomical structure of the complex root canal system often result in furcal perforation, ledge, canal transportation, strip perforation, root perforation, instrument separation, voids in the obturation, or underfilling or overfilling of the obturation, which leads to reinfection of the tooth. The application of microrobotic tools reduces teeth reinfection and promotes more accurate, minimally invasive root canal treatment [54]. It is not easy to distinguish root canal calcification from the naked eye. Microrobotic tools can magnify the difference in the color and texture between calcified and normal dentin, which provides powerful help for dredging small calcified root canals, as shown in Figures 3(i) and 3(j), taking the C-shaped root canal as an example of root canal variation. Because of the tortuous structure of the C-shaped root canal, pulp tissue or other debris will remain in the isthmus of the root canal during clinical root canal preparation, causing reinfection of the affected tooth and leading to the failure of root canal treatments [55]. In addition, C-shaped root canals are also prone to root canal perforation during preparation. As a serious complication, perforation, especially through the alveolar ridge, can cause abnormal communication between the pulp cavity and the periodontal tissue, which destroys the periodontal tissue, as shown in Figures 3(k) and 3(l). The microscope can not only illuminate the affected area but also allow the doctor to see the direction of the root canal more clearly based on the different colors of the root canal dentin and root canal perioral dentin, which is conducive to the good preparation of ultrasonic washing, chemical preparation, and other preparation techniques. Using microrobotic tools can not only reduce the occurrence of iatrogenic traumas such as furcal perforation, ledge, canal transportation, strip perforation, root perforation, instrument separation, voids in the obturation, or underfilling or overfilling of the obturation but can also be remedied when trauma occurs [56].

*(3) Root Canal Filling*. The analysis of the failure case indicated that the most common cause of failure was a leaky canal (30.4%), followed by a missing canal (19.7%), underfilling (14.2%), anatomical complexity (8.7%), overfilling (3.0%), iatrogenic problems (2.8%), apical calculus (1.8%), and apical cracks (1.2%) [57]. One of the primary causes of failed root canal treatment is an inadequate filling of the root canal system, in other words, the presence of gaps between the root canal filling material and the dentinal walls. Figures 3(m) and 3(n) show incorrect root canal filling.

*(4) Removal of Obstructions in the Root Canal*. In root canal therapy, the original pulp is usually removed. If the instrument is separated and stuck in the middle of the root canal, doctors should remove the separated instrument from the root canal. Similar to the situation faced by root canal preparation, removing obstructions in the root canal becomes difficult due to the complex anatomy of root canal systems [58]. Clinically, microscopy is usually combined with ultrasound technology to prepare teeth for root canal retreatments. Under the microscope, the doctor can clearly distinguish the separation device, the plasticizing fluid, and the adhesive between the dowel and the root canal wall and then remove it by the ultrasound technique [59]. Figure 3(p) shows the separation device in the root canal.

#### 3.1.3. Endodontic Microsurgery and Development of Robot-Assisted Endodontic Therapy

Traditional periradicular surgery includes periradicular curettage, apicoectomy, and retrograde filling [60]. Microrobotic tools can make the operation more precise and more minimally invasive. In microsurgery, the microscope presents periapical lesions, which helps to accurately locate the root apex, collateral root canals, intercanal isthmus, missing root canals, and other structures, improves the surgical access and visibility of the apical area, and weakens the trauma caused by the operation at the same time. All of the above factors achieve the effect of precise preparation and tightly sealing the root apex, increasing the success rate of traditional apical surgery from 59.0%–71.9% to 91.7%–94.0% [61]. Iwai et al. showed in vitro training in endoscopic periradicular surgery using a printed three-dimensional model [62]. Garcia et al. reported a case of apical surgery of a maxillary molar by endoscopy [63]. A study compared microscopes versus endoscopes in root-end management. Researchers reported that microscopes and endoscopes were effective, and above 90% successful healing was achieved [20].  Figure 4 shows a case of the periradicular surgery conducted by the microscope and the endoscope. In addition to the use of robotic and microrobotic tools, robots and microrobots are also used in endodontic therapy. A robot was reported as a “vending machine” to provide the clinician with the required root canal therapy instruments during the procedure [64]. Janet Dong et al. reported an endodontic microrobot to complete root canal treatment automatically. However, this paper only described the preliminary development, including specifications and requirements, mechanical design, and controller systems [65]. In 2010, his further study described the design of a *Z* axis actuator and tool quick change assembly in the micromachine for root canal treatment. However, further modification of the design may be needed after testing, and there are no longer any reports [66]. Microrobotic tools are now contributing to minimally invasive treatment rather than robotic treatment. Microrobots are the future direction of robot-assisted endodontic therapy. A recently published report suggested that a microrobot with catalytic ability could destroy the oral biofilm in the root canal and analyze the robot system in the laboratory.  Figure 5 shows the CARs to act as a microrobot. In addition, the researchers explained the application of these robot systems in other applications, including the prevention of peri-implant infection or dental caries [67]. The use of robots in endodontics is very few. However, endodontic therapy is the most difficult to operate and needs the most robotic and microrobotic tools. Therefore, most of the context here is spent elaborating on the needs of endodontic doctors.

### 3.2. Robotic and Microrobotic Tools in Periodontology

We can define periodontal disease as an infectious bacterial disease resulting in an attack of tooth-supporting structures: bone, gums, cement, and the ligament system that anchors the tooth to the bone, including epithelial attachment [68]. This disease presents various degrees of severity, rates of progression, and responses to treatments. The most common means to diagnose periodontal disease is visual examination, assisted by a periodontal probe and radiographs. The periodontal probe gives a quantified reading of periodontal tissue damage, and the radiographs allow visualization of some of the structures not visible by direct vision, especially the interproximal bone [69]. In addition to subgingival plaque, subgingival calculus will also affect periodontal calculus, as a foreign body in the mouth will continue to stimulate and compress the periodontal calculus and promote the production or intensification of local periodontal tissue inflammation. Therefore, the removal of subgingival plaque and calculus has become the basis of periodontal treatment. Since the removal target is under the gums, the accuracy of periodontal surgery is required. Shanelec et al. found that dental calculus and inflammation coverage was significantly reduced after microscopy was used [70]. In summary, it is fully proven that microscope use, or magnification of the field of view, has positive effects on periodontal treatment.

In periodontal surgery, whether using sound waves, ultrasound, or manual techniques, it will inevitably have a destructive effect on the tooth's structure, causing deviations in operation. The application of magnifying equipment such as microscopes in periodontal treatment reduces this deviation, improves the accuracy of periodontal surgery, reduces periodontal surgery wounds, shortens the wound healing time, and reduces the formation of postoperative scars. Robotic and microrobotic tools have a significant effect on the transplantation of periodontal soft tissue flaps [71]. Dental endoscopes have already been used in periodontology and may provide additional benefits for calculus removal compared with traditional SRP [72].

Few robots are used in periodontology. Robots are only used to help clean teeth. Similarly, Ernst et al. developed a robot system to simulate the change in 3D brushing motion over time [73]. In vitro, experimental results show that the robot system can show repeatable significant differences in the cleaning effect of electric toothbrushes.

### 3.3. Robotic and Microrobotic Tools in Oral and Maxillofacial Surgery

Oral and maxillofacial surgery involves treatment of oral organs (teeth, alveolar bone, lips, cheeks, tongue, palate, pharynx, etc.), facial soft tissues, maxillofacial bones (upper jaw, mandible, cheekbone, etc.), surgical treatment of the temporomandibular joint, salivary glands, etc. [74–78]. The pathological section of surgical tumor resection was where the microscope was first used. Initially, microscopy was mainly used for postoperative observation of tumors or cysts. After the development of microsurgery technology, robotic and microrobotic tools have been widely used in oral surgery clinics: oral microsuturing can be used to suture small tissues such as blood vessels finely; oral microdiagnosis can identify cancerous tissues and cyst walls; oral microscopic resection of tumors can accurately locate the resection site and reduce trauma; oral microscopic pathological examination of the surgical margins ensures clean resection [79]. With the magnification of the field, robotic and microrobotic tools help doctors locate the lesion accurately and significantly reduce the wound area [80].

The application of microsurgery technology improves the success rate of free tissue transplantation into the recipient area. Surgeons can effectively repair maxillofacial injuries based on free transplantation, according to different vascularized body tissues. Oral and maxillofacial repair and reconstruction involve free tissue transplantation that requires anastomosis of blood vessels. Treatment should consider not only the prospect of tissue recovery but also aesthetics. According to research, the success rate of maxillofacial repair under microsurgery technology has significantly improved, and the incidence of complications has been reduced [81, 82]. Dentists can also use robotic and microrobotic tools for nerve repair, which is challenging to operate without magnification [83]. Endoscopic surgery of the temporomandibular joint is becoming an important research direction in treating the temporomandibular joint [84, 85].

In summary, the application and development of dental surgery microscopes promote the minimization of iatrogenic damage in surgical treatment, the minimization of medical costs, and the maximization of patient rehabilitation. Robots are also used in oral and maxillofacial surgery. In 2009, the US Food and Drug Administration approved the Da Vinci system for oral treatment of some malignant diseases [86] and all nonmalignant lesions of the oropharynx, even at the bottom of the throat and tongue. Robot-assisted surgery can also provide good local control in the treatment of low-risk oral squamous cell carcinoma [87]. The oral application of this part is similar to the application of robots in surgery.

### 3.4. Robotic and Microrobotic Tools in Oral Medicine

There are many kinds of oral mucosal diseases with various causes. The diagnosis of mucosal diseases usually requires the observation of robotic and microrobotic tools. Doctors often need to take a biopsy or smear observation to diagnose mucosal disease. The mucosal disease can develop into cancer. After pathological examination, the cells need to be observed and confirmed by robotic and microrobotic tools [88–90]. The most important thing of mucosal diseases is the diagnosis, and the most common treatment is drug treatment. Therefore, microscopes and endoscopes can help diagnosis, but few robots appear to help treatment.

### 3.5. Robotic and Microrobotic Tools in Prosthodontics

The highest goal of prosthodontics is to make false teeth that mix spurious with genuine teeth. The most common products of prosthodontics are crowns, veneers, and inlays [91, 92]. If you want a natural last appearance of dentures, you need high polishing, good preparation. The finish line is the place where the prosthesis and the natural tooth are connected. If preparing the finish line is not fine enough, it will cause a series of problems and damage the stable environment in the oral cavity. The rough finish line means an insufficient connection between the prosthesis and the natural teeth, even a gap. Food residue and bacteria will accumulate in the gap, causing secondary caries. Imperfect shoulders can also lead to a protruding foreign body at the edge of the crown, which can stimulate the gums and cause complications such as gingival inflammation and bleeding [93]. Therefore, a continuous, clear, precise, smooth finish line will help improve the accuracy of the impression, significantly improving the adhesion between the final restoration and the preparation. It will also help to avoid stimulating periodontal soft tissue and prevent complications such as secondary caries caused by edge microleakage and loss of periodontal attachment and create a long-term stable oral environment. To monitor the effect of finish line preparation in real time, in addition to visual observation, a dental operating microscope can be used clinically. However, in recent years, after the concept of precise preparation was put forward, an increasing number of dentists began to pursue higher-precision preparation methods. Microscope operations gradually emerged in dental restorations: preliminary tooth preparation at low magnification; the rough parts are enlarged and finely polished one by one; polishing is carried out at high magnification to remove the fine cracks on the tooth preparation, forming a smooth tooth preparation. Dentists evaluated the accuracy of the impression with a microscope.

Most of the articles on prosthodontic robots are not exceeding the level of proof of concept, including the tooth-arrangement robots [94]. A tooth preparation robot system was invented and showed its clinical potential [95]. The report shows good results, but its results have not been verified in clinical settings thus far.

### 3.6. Robotic and Microrobotic Tools in Implant Dentistry

Robotic and microrobotic tools are widely used in implant dentistry. Limited by the patients' maxillary sinus bone quality, maxillary sinus lifting will be used in implant surgery to increase the success rate of implant surgery. Nevertheless, maxillary sinus lifting is not performed under direct vision, which may easily cause perforation of the sinus mucosa, leading to maxillary sinusitis. Endoscopic-assisted maxillary sinus lifting is a maxillary sinus lifting technique under endoscopic monitoring [22]. The doctor can use the endoscope inserted into the sinus through the canine fossa on the nasal side of the maxillary sinus to monitor the integrity of the maxillary sinus mucosa in real time during maxillary sinus lifting to better control the lifting height and the position of the graft material and provide timely feedback and rescue when perforation occurs, which dramatically reduces iatrogenic trauma and perforation probability.

For implant dentistry, robotic surgery is already a reality. In 2002, Boesecke et al. reported the first study of robot-assisted dental implantation to minimize error [96]. In 2013, controlled and accurate drilling was achieved by a new robotic system [97]. In 2015, a 3-DOF robot which can detect and modulate the handpiece to ensure the accuracy of implantation was released [98]. The dental implant robots are not exceeding the level of proof of concept until 2017. In 2017, the Neocis Yomi robotic device (USA) became the world's first FDA-approved computer navigation robot system [99]. In 2017, The Autonomous Dental Implant Robot System was invented by the Fourth Military Medical University Hospital and Peking University [86]. The Autonomous Dental Implant Robotic System was approved by the National Medical Products Administration (NMPA) and clinical trials were under way. The robot system aims to prevent surgical errors and solve the problem of the lack of high-quality dentists in China.

### 3.7. Robotic and Microrobotic Tools in Dental Photomicrography and Oral Radiology

The initial application of dental photography in the clinic is mainly to record the anatomical shape and color characteristics of the soft and hard tissues of the oral cavity and maxillofacial region to provide support for doctors' clinical diagnosis, case records, formulation of treatment plans, and prognosis, effectively facilitating communication with doctors, patients, and colleagues. With the development of technology and the progress of the times, dental clinical operation is gradually refined and modernized. The demand for recording accurate dental operations has gradually increased, and dental photomicrography has also emerged. Compared with traditional photography, dental photomicrography is more suitable for shooting small parts such as root canals. It records the tiny parts of teeth more precisely and takes efficient, serial, and high-definition photos of the diagnosis and treatment process without affecting the treatment process [100].

It is generally believed that oral radiologists can penetrate almost all aspects of oral teeth in a minimally invasive manner. Burdea et al. designed a robot system for tooth subtraction photography, using a 6-DOF position sensor, and proposed a robot arm with an X-ray source [101].

## 4. Strengths and Weaknesses

The strengths and weaknesses of robotic and microrobotic tools are summarized in Table 1.

### 4.1. Strengths

1. Most robotic and microrobotic tools have a lighting system.
2. The naked eye resolution is only 0.2 mm, while the dental operating microscope can be magnified 2–30 times. The limit resolution of the dental operating microscope can reach 0.006 mm, significantly improving human eye resolution and obtaining more visual information to help with minimally invasive treatments [102]. In clinical operation, when adjusting magnification, there is no need to change the location of the microscope, and the stability of the field is good.
3. Ergonomics is essential to the health of dentists. The investigation shows that more than 70% of clinicians whose long-term head anteversion angle is greater than 20 degrees will suffer from shoulder and neck pain. More than 85% of the clinicians who did not wear loupes had head anteversion greater than 30 degrees [103]. In addition, the use of a dental operating microscope can also achieve improved ergonomics at other levels. Using a dental operating microscope, the eyepiece and observation object distance are relatively stable, reducing unnecessary adjustment [104].
4. Doctors and patients can maintain a relatively safe distance, reducing the risk of saliva and blood infection. The dental operating microscope can be equipped with an assistant mirror to facilitate the cooperation of the assistant during the operation of the microsurgery [105]. Skilled dentists and assistants can achieve more efficiency.
5. Robotic and microrobotic tools can be equipped with a camera or a video camera and other image acquisition devices to realize real-time recording of the treatment process. Image data are conducive to doctor-patient communication so that patients can participate in developing treatment plans. It is also conducive to dental clinical teaching demonstration.
6. The realization of virtual reality is expected to realize remote diagnosis and treatment [37].

### 4.2. Weaknesses

1. The cost of robotic and microrobotic tools is high
2. Robotic and microrobotic tools are precision instruments that need professional maintenance and regular maintenance
3. Because of its use and operation complexity, operators and their assistants need special clinical operation training before use and need a certain adaptation period
4. Robotic and microrobotic tools lack the operating devices that eventually become robots and microrobots

## 5. Conclusion and Outlook

Dentistry is moving toward a new world of robot-assisted and data-driven medicine. Judging from the dependence of stomatology on tools, stomatologists need practical tools very much. With the increasing use of robots and microrobot tools in fields other than endodontics, their importance in dental clinics has been gradually recognized. They amplify nuances that the human eye cannot see and the prospect of precise medical treatment. It is crucial for complex root canal exploration, cancer tissue excision, and other oral cavity procedures. In specific ways, they broaden the scope of oral clinics, promote the future of oral clinics, and strive to balance iatrogenic injuries and the rehabilitation of the afflicted region. Robotic and microrobotic tools provide several advantages in dental clinics. Nevertheless, the main drawbacks are the lack of cost-effectiveness produced by the high cost of microscopes and the technical sensitivity created by the difficulty of operating the microscope. We expect that the widespread use of microrobotic instruments will enable the implementation of an oral treatment regimen. Virtual reality robotic and microrobotic tool skill training will be accomplished soon. The reality is that robots are not widely used in dentistry. Robots may need to learn from the functions of these tools. What limits the development of dental robots? First, the development and use of robots are expensive. Second, robots systems are complex systems. At present, dental robots only do some simple work, but these microscopic tools can help doctors complete complex work, which may be one reason. Dentists' acceptance of robots depends largely on demand. On the other hand, the acceptance of robots to patients has not been improved, and patients are not ready for robotic surgery. In addition, the use of robots must rely on the critical input of data. However, with the development of the times, these problems will eventually be overcome. Oral treatment programs also include artificial intelligence, lowering the technical threshold for application and attaining clinical popularization. It is believed that in the near future, robotic microscopes and robotic endoscopes will spring up and occupy the market. This will also open the prelude for the robot to finally complete the treatment independently.

## Figures and Tables

**Figure 1:** Robotic and microrobotic tools for dental treatments. (a) An operating microscope. (b) An endoscope. (c) A robotic manipulator of a robotic endoscopic system. Copyright 2019, Hindawi.

**Figure 2:** An endoscopic system. (a) A schematic diagram of an endoscopic system. (b) Cross-sectional schematic diagram of the probe.

**Figure 3:** Photos in the endodontics therapy. (a) A decayed tooth. (b, c) A cracked tooth. (d) Deep caries infected pulp. (e) A tooth with P2. (f, g) A tooth with MB2. (h) A tooth with ML2. (i, j) Calcification of pulp cavity. (k, l) Destruction of pulp chamber bottom. (m, n) Root filling is incorrect. (o, p) Broken needle in root canal.

**Figure 4:** The periapical microsurgery with an endoscope and microscope.of two upper central incisors. (a) Preoperative clinical view. (b) X-ray showing low-density images around the end of roots. (c) CBCT showing the destruction of the buccal cortical layer of the left upper incisor. (d) Incision. (e) Raising of the full-thickness mucoperiosteal flap (f) Ostectomy and curettage of the periapical lesions. (g) Endoscopic view of the right upper incisor. (h) Endoscopic view of the left upper incisor. (i) Clinical view of the removal of the old filler material. (j) Endoscopic view of the right upper incisor after removal of the old filler material. (k) Endoscopic view of the left upper incisor after removal of the old filler material. (l) Clinical view of filling with MTA. (m) Endoscopic view of the right upper incisor after filling with MTA. (n) Endoscopic view of the left upper incisor after filling with MTA. (o) Bone transplantation with bone graft. (p) Suture the operation area. (q) 7 days after the operation. (r) 1 year after the operation. (s) X-ray showing good bone healing after 1 year. (t) After tooth preparation with the BOPT approach. (u) Occlusal view. (v) After installation of the provisional crowns. (w) After cementing the definitive crowns. (x) The smiling photo. Copyright 2020, Hindawi.

**Figure 5:** A magnetic microrobot for catalytic biofilm degradation.

**Table 1:** Strengths and weaknesses of robotic and microrobotic tools.

Robotic and microrobotic tools	
Strengths	Weaknesses
Always a lighting system	Increase the cost
Appropriate magnification and more minimally invasive	Professional maintenance and regular maintenance
Reasonable ergonomic design	Lack the operating devices
More secure and efficiency	Special clinical operation training
Data record-keeping and teaching	
The realization of virtual reality	

## Data Availability

No data were used to support this study.
